# A Novel Framework Based on Deep Learning and ANOVA Feature Selection Method for Diagnosis of COVID-19 Cases from Chest X-Ray Images

**DOI:** 10.1155/2022/4694567

**Published:** 2022-01-07

**Authors:** Hamid Nasiri, Seyed Ali Alavi

**Affiliations:** ^1^Department of Computer Engineering, Amirkabir University of Technology, Tehran, Iran; ^2^Electrical and Computer Engineering Department, Semnan University, Semnan, Iran

## Abstract

*Background and Objective*. The new coronavirus disease (known as COVID-19) was first identified in Wuhan and quickly spread worldwide, wreaking havoc on the economy and people's everyday lives. As the number of COVID-19 cases is rapidly increasing, a reliable detection technique is needed to identify affected individuals and care for them in the early stages of COVID-19 and reduce the virus's transmission. The most accessible method for COVID-19 identification is Reverse Transcriptase-Polymerase Chain Reaction (RT-PCR); however, it is time-consuming and has false-negative results. These limitations encouraged us to propose a novel framework based on deep learning that can aid radiologists in diagnosing COVID-19 cases from chest X-ray images. *Methods*. In this paper, a pretrained network, DenseNet169, was employed to extract features from X-ray images. Features were chosen by a feature selection method, i.e., analysis of variance (ANOVA), to reduce computations and time complexity while overcoming the curse of dimensionality to improve accuracy. Finally, selected features were classified by the eXtreme Gradient Boosting (XGBoost). The ChestX-ray8 dataset was employed to train and evaluate the proposed method. *Results and Conclusion*. The proposed method reached 98.72% accuracy for two-class classification (COVID-19, No-findings) and 92% accuracy for multiclass classification (COVID-19, No-findings, and Pneumonia). The proposed method's precision, recall, and specificity rates on two-class classification were 99.21%, 93.33%, and 100%, respectively. Also, the proposed method achieved 94.07% precision, 88.46% recall, and 100% specificity for multiclass classification. The experimental results show that the proposed framework outperforms other methods and can be helpful for radiologists in the diagnosis of COVID-19 cases.

## 1. Introduction

The new Coronavirus disease, also known as COVID-19, was initially discovered in Wuhan, China, in December 2019 [1]. COVID-19 is the name of the disease, and SARS-CoV-2 is the name of the virus. This novel infection spread from Wuhan to a large portion of China in less than 30 days [2]. On 11 March 2021, the World Health Organization (WHO) declared the outbreak a pandemic [3, 4]. Since 19 November 2020, the COVID-19 pandemic has had a detrimental effect on the world, with approximately 219,456,675 confirmed cases and 4,547,782 deaths reported till 27 September 2021; in addition, nearly 7.7 million workers have lost their jobs in America [5]. The global recession and closure of schools and institutions worldwide have significantly impacted mental and physical health [3]. The majority of Coronaviruses infect animals; however, due to their zoonotic nature, they can infect humans [6]. As a result, it can potentially infect human airway cells, leading to pneumonia, severe respiratory infections, renal failure, and even death. Fever, cough, sore throat, headache, weariness, muscle soreness, and shortness of breath are common COVID-19 symptoms [7].

Vivid screening of infected individuals allows them to be isolated and treated and is a crucial and essential step in combating COVID-19 [1]. Reverse Transcriptase-Polymerase Chain Reaction (RT-PCR) testing, which can identify SARS-CoV-2 RNA from respiratory material, is the most common technique for detecting COVID-19 patients [8]. It requires specialized materials and equipment that are not readily available; because of the large number of false-negative results, it takes at least 12 hours, which is inconvenient considering that positive COVID-19 patients should be identified and followed up on as soon as possible [4, 9, 10]. Chest CT scan is another option for detecting the disease, which is more accurate than RT-PCR; For instance, 75% of negative RT-PCR samples had positive results on chest CT scans [11]. CT scans have several drawbacks, including image collection time, related cost, and CT equipment availability [12]. When compared to CT scans, X-ray images are less expensive and more easily available [13]. As a result, the focus of the research is only on the use of X-ray imaging as a screening tool for COVID-19 patients.

Researchers discovered that COVID-19 patients' lungs contain visual markings such as ground-glass opacities—hazy darker areas that may distinguish COVID-19-infected individuals from noninfected patients [14, 15]. However, due to the limitations of experts, time constraints, and the irreversible consequences of misdiagnosis [6], it is crucial to discover a different approach to get faster and more reliable outcomes. The technological advancements facilitate the process of diagnosing the diseases; in other words, the widespread use of Artificial Intelligence (AI) [16], mainly its areas such as machine learning and deep learning, is extremely constructive, and researchers have made significant use of AI and deep learning in various medical areas [4, 17]. Convolutional neural network (CNN) architecture is one of the most prominent deep learning techniques in the medical imaging field, with outstanding results [18].

Pretrained neural networks are used in this paper, which is one of the most recent techniques. Using easily accessible pretrained models, the proposed method extracts features from X-ray images. We utilize one of the feature selection methods in the second phase to acquire an appropriate number of features for classification. Finally, we use the eXtreme Gradient Boosting (XGBoost) classifier to classify the specified features. A preprint of this paper has previously been published [19]. The major contributions of this paper are summarized as follows:

1. We used an easily accessible pretrained model, DenseNet169 for feature extraction, and XGBoost for classification as a brand-new approach.
2. Using a feature selection approach, i.e., analysis of variance (ANOVA), improves prediction performance and obtains an adequate number of features for classification and reduces complexity.
3. Effectiveness of the proposed method is evaluated using the ChestX-ray8 dataset. The experimental results show that the proposed method effectively classifies COVID-19 cases, and the classification accuracy is considerably increased.

The rest of the paper is organized as follows.  Section 2 describes related works. In Section 3, used materials and methods will be presented. In Section 4, the experimental results are reported and analyzed. Finally, Section 5 will present a summary of the findings and conclusions.

## 2. Related Works

Researchers worldwide are now fighting against COVID-19; using radiological imaging and deep learning has made significant progress in this approach. Wang et al. [8] developed COVID-Net, a deep model for COVID-19 detection that categorized normal, non-COVID-19 pneumonia, and COVID-19 classes with 92.4 percent accuracy. Apostolopoulos and Mpesiena [20] applied transfer learning and employed COVID-19, healthy, and pneumonia X-ray images to develop their model. Ozturk et al. [6] proposed using the DarkNet model to build a deep network. This model contains 17 convolution layers and utilizes the Leaky ReLU activation function. The mentioned model was 98.08% accurate for binary classes, and for multiclass cases, it was 87.02% accurate. Nasiri and Hasani [21] employed DenseNet169 to extract features from X-ray images and used XGBoost for classification; they gained 98.24% and 89.70% in binary and multiclass classification, respectively.

Qaid et al. [22] applied deep and transfer learning approaches to build reliable, general, and robust models for identifying COVID-19. Abdulkareem and Mpesiena [23] proposed a model to detect COVID-19 cases in smart hospitals utilizing machine learning and the Internet of Things. Chen and Rezaei [24] proposed a method for extracting 18 different features from X-ray images. The minimal features are chosen using a metaheuristic algorithm called the Archimedes optimization to reduce the approach's complexity. Khorami et al. [25] proposed a method for extracting a combination of gray-level co-occurrence matrix (GLCM) and Discrete Wavelet Transform (DWT) features from X-ray images, followed by classification of the images using an improved CNN model, based on the Red Fox Optimization algorithm. Waheed et al. [26] developed an Auxiliary Classifier Generative Adversarial Network (ACGAN)-based model called CovidGAN to create synthetic X-ray images and improve the accuracy of COVID-19 classification.

Sethy et al. [27] devised an in-depth feature combined support vector machine (SVM) based method for detecting coronavirus-infected individuals using X-ray images. SVM is examined for COVID-19 identification utilizing the deep features of 13 different CNN models. Fareed Ahmad et al. [28] utilized X-ray images for training deep CNN models like MobileNet, ResNet50, and InceptionV3 with a variety of options, including starting from scratch, fine-tuning with learned weights of all layers, and fine-tuning with learned weights and augmentation. Abbas et al. [29] verified a deep CNN termed Decompose, Transfer, and Compose (DeTraC) for COVID-19 chest X-ray image classification. Wang et al. [30] presented the Parallel Channel Attention Feature Fusion Module (PCAF) and a new convolutional neural network MCFF-Net based on PCAF. The network uses three classifiers to boost recognition efficiency: 1-FC, GAP-FC, and Conv1-GAP. Ucar and Korkmaz [31] developed the SqueezeNet that goes toward its light network design, is optimized for the COVID-19 detection with the Bayesian optimization additive.

Additionally, Kang et al. [32] presented a transfer learning model that handles a dataset of COVID-19-infected patients' CT images. They achieved a test accuracy of 79.3%. Khan et al. [1] represented CoroNet, a deep CNN model for automatic diagnosing of COVID-19 from chest X-ray images. The proposed model is built on the Xception architecture. Narin et al. [33] proposed five models for diagnosing people with pneumonia and coronavirus using X-ray images.

Similarly, He et al. [34] created a deep learning method to categorize COVID-19. They scanned 746 CT images, 349 of which were of infected patients and 397 of healthy people. The Self-Trans technique is proposed in this approach, which combines contrastive self-supervised learning with transfer learning to gain unbiased and robust feature representations while avoiding overfitting, resulting in a 94% accuracy rate. Xu et al. [35] applied deep learning techniques to create an early screening model to discriminate COVID-19 from influenza-A viral pneumonia and healthy cases using chest CT scans. Hemdan et al. [36] used 50 validated chest X-ray images and 25 confirmed positive COVID-19 cases and developed the COVIDX-Net, which incorporates seven distinct architectures of deep convolutional neural network models, such as VGG19 as well as the second version of Google MobileNet. Minaee et al. [37] used publicly available datasets to build a dataset of 5000 chest X-rays. A board-certified radiologist discovered images that showed the existence of the COVID-19 virus. Four prominent convolutional neural networks were trained to detect COVID-19 disease using transfer learning.

## 3. Materials and Methods

The proposed method employs the DenseNet169 deep neural network, the ANOVA feature selection method, and the XGBoost algorithm, which will be discussed in the following section.

### 3.1. DenseNet169

A CNN's overall architecture is composed of two core parts: a feature extractor and a classifier. Convolution and pooling layers are the two essential layers of CNN architecture. Each node in the convolution layer extracts features from the input images by performing a convolution operation on the input nodes. The max-pooling layer abstracts the features by averaging or calculating the maximum value of input nodes [38, 39]. DenseNet is a highly supervised network containing a 5-layer dense block with a *k* = 4 rate of growth and the standard ResNet structure. Each layer's output in a DenseNet dense block includes the output of all previous layers, incorporating both low-level and high-level features of the input image, making it suitable for object detection [40]. The ILSVRC 2012 classification dataset used for training DenseNet contains 1,000 classes and 1.2 million images. The dataset images were cropped with the size of 224 × 224 before using as input for DenseNet. DenseNet presented a new connectivity pattern that introduced direct connections from any layer to all the following layers to further improve information flow across layers [41]. In DenseNet, the *l* th layer takes all feature maps *x*_0_, *x*_1_, *x*_2_,…, *x*_*l*−1_ from the preceding layers as input, which is described by

(1) $$\begin{array}{c} x_{1}=H_{1}\left(\left[x_{0},x_{1},x_{2},\ldots ,x_{l-1}\right]\right), \end{array}$$

where *H*_*l*_(·) is a singular tensor and [*x*_0_, *x*_1_, *x*_2_,…, *x*_*l*−1_] is the concatenated features from *l* − 1 layers. To preserve the feature-map size constant, each side of the inputs is zero-padded by one pixel for convolutional layers with kernel size 3 × 3. DenseNet employed 1 × 1 convolution and 2 × 2 average pooling as transition layers between adjoining dense blocks. A global average pooling is conducted at the end of the last dense block, and then a Softmax classifier is connected. In the three dense blocks, the feature-map sizes are 32 × 32, 16 × 16, and 8 × 8, respectively. On five distinct competitive benchmarks, this innovative architecture reached state-of-the-art accuracy for recognizing the objects [38, 41].

### 3.2. Analysis of Variance Feature Selection

New issues develop as a result of the creation of large datasets. Consequently, reliable and unique feature selection approaches are required [42]. Feature selection can assist with data visualization and understanding and minimize measurement and storage needs, training and utilization times, and overcoming the curse of dimensionality to enhance prediction performance [42, 43]. ANOVA is a well-known statistical approach for comparing several independent means [44]. The ANOVA approach ranks features by calculating the ratio of variances between and within groups [45].

The ratio indicates how strongly the *λ* th feature is linked to the group variables. The following equation is used to calculate the ratio *F* value of *λ* th g-gap dipeptide in two benchmark datasets:

(2) $$\begin{array}{c} F\left(\lambda \right)=\frac{s_{B}^{2}\left(\lambda \right)}{s_{W}^{2}\left(\lambda \right)}, \end{array}$$

where *s*_*B*_^2^(*λ*) and *s*_*W*_^2^(*λ*) are the sample variance between groups (also known as Mean Square Between, MSB) and within groups (also known as Mean Square Within, MSW), respectively, and can be calculated as

(3) $$\begin{array}{c} s_{B}^{2}\left(\lambda \right)=\sum_{i=1}^{K}n_{i}\frac{{\left(\left(\sum_{j=1}^{n_{i}}f_{ij}\left(\lambda \right)/n_{i}\right)-\left(\sum_{i=1}^{K}\sum_{j=1}^{n_{i}}f_{ij}\left(\lambda \right)/\sum_{i=1}^{K}n_{i}\right)\right)}^{2}}{\text{d}f_{B}}, \end{array}$$

(4) $$\begin{array}{c} s_{W}^{2}\left(\lambda \right)=\sum_{i=1}^{K}\sum_{j=1}^{n_{i}}\frac{{\left(f_{ij}\left(\lambda \right)-\left(\sum_{i=1}^{K}\sum_{j=1}^{n_{i}}f_{ij}\left(\lambda \right)/\sum_{i=1}^{K}n_{i}\right)\right)}^{2}}{\text{d}f_{W}}. \end{array}$$

The degrees of freedom for MSB and MSW are d*f*_*B*_=*K* − 1 and *df*_*W*_=*N* − *K*, respectively. The number of groups and the total number of samples are represented by *K* and *N*, respectively. The frequency of the *λ* th feature in the *j* th sample in the *i* th group is denoted by *f*_*ij*_(*λ*). The number of samples in the *i* th group is denoted by *n*_*i*_ [46].

### 3.3. Extreme Gradient Boosting (XGBoost)

Chen and Guestrin proposed an efficient and scalable variation of the Gradient Boosting algorithm called XGBoost. XGBoost has been widely employed by data scientists recently, and it had desirable results in a wide range of machine learning competitions [47, 48]. In certain ways, XGBoost differs from Gradient Boosted Decision Trees (GBDT). First of all, the GBDT algorithm only employs a first-order Taylor expansion, whereas XGBoost augments the loss function with a second-order Taylor expansion. Secondly, the objective function uses normalization to prevent overfitting and reduce the method's complexity [49–51]. Third, XGBoost is extremely adaptable, allowing users to create their own optimization objectives and evaluation criteria. Nevertheless, by establishing class weight and using Area Under the Curve (AUC) as an assessment criterion, the XGBoost classifier can handle unbalanced training data efficiently. In summary, XGBoost is a scalable and flexible tree structure improvement model that can manage sparse data, enhance algorithm speed, and minimize computing time and memory for large-scale data [52].

Formally, the XGBoost algorithm can be described as follows.

Given a training dataset of *n* samples *T*={(**x**_1_, *y*_1_), (**x**_2_, *y*_2_),…, (**x**_*n*_, *y*_*n*_)}**x**_*i*_ ∈ *ℝ*^*m*^*y*_*i*_ ∈ *ℝ*, the objective function can be defined by

(5) $$\begin{array}{c} \text{obj}\left(\theta \right)=\sum_{i}^{n}l\left(y_{i},{\hat{y}}_{i}\right)+\sum_{t=1}^{T}\Omega \left(f_{t}\right), \end{array}$$

where $l\left(y_{i},{\hat{y}}_{i}\right)$ measures the difference between the target *y*_*i*_ and the prediction ${\hat{y}}_{i}$ and *f*_*t*_ denotes the prediction score of *t* th tree [53]. Ω(*f*_*t*_) represents the regularization term, which control the model's complexity to avoid overfitting [50]. The estimated loss function can be computed based on Taylor expansion of the objective function:

(6) $$\begin{array}{c} L^{\left(t\right)}≃\sum_{i=1}^{k}\left[l\left(y_{i},{\hat{y}}^{\left(t-1\right)}\right)+g_{i}f_{t}\left(x_{i}\right)+\frac{1}{2}h_{i}f_{t}^{2}\left(x_{i}\right)\right]+\Omega \left(f_{t}\right), \end{array}$$

where $g_{i}=\partial_{{\hat{y}}^{\left(t-1\right)}}l\left(y_{i},{\hat{y}}^{\left(t-1\right)}\right)$ denotes each sample's first derivative and $h_{i}=\partial_{{\hat{y}}^{\left(t-1\right)}}^{2}l\left(y_{i},{\hat{y}}^{\left(t-1\right)}\right)$ denotes each sample's second derivative. The first and second derivatives of each sample are all that the loss function requires [54].

### 3.4. Proposed Method

In this study, preprocessing methods were employed on the dataset, including label encoder for classes and normalization on images. As a result, less redundant data are given as the input to the network. Deeply influenced by the brain's structure, deep learning as a subfield of machine learning has emerged. In medical image processing, as in many other areas, deep learning approaches have demonstrated excellent results in past years [33]. ImageNet is a dataset of millions of images organized into 1000 categories when it comes to image processing. The next step was to apply several pretrained models that were trained based on this dataset. DenseNet169 had the best performance among those models, so it was selected as the feature extractor in the proposed method. The X-ray dataset images were scaled at a fixed size of 224 × 224 pixels, the DenseNet169 input size.

The final layer of the DenseNet169 network, which was used to predict ImageNet dataset labels, was eliminated. Global average pooling, a pooling method designed to substitute fully connected layers in classical CNNs, was added in the final layer of the network. One of the benefits of global average pooling is that there are no parameters to adjust in this layer; therefore, no training is needed. Additionally, because global average pooling sums up the dimensional information, it is more robust to spatial translations of the input [55]. The X-ray images were given to the network to extract features from DenseNet169, and 1664 features were extracted as a result.

When a learning model is given many features and few samples, it is likely to overfit, causing its performance to degrade. Among researchers, feature selection is a widely used strategy for reducing dimensionality [56]. In order to reduce the classification time and increase the classifier performance, the ANOVA feature selection method was employed to reduce the number of features. Thus, the range of 50 to 500 features was applied to select the best number of features for classification (using validation set). Finally, the selected features were given to the XGBoost to detect COVID-19.  Figure 1 shows the general framework of the proposed method.

## 4. Results and Discussion

Several performance metrics such as precision, recall, specificity, and *F*_1_-Score, as well as accuracy, were utilized to evaluate several deep learning models with the proposed methodology because accuracy alone cannot evaluate a model's usefulness [57]. Accuracy is the ratio of the number of correctly predicted samples to the total number of samples. The following equation can be used to calculate accuracy:

(7) $$\begin{array}{c} \text{accuracy}=\frac{\text{TP}+\text{TN}}{\text{Total}}, \end{array}$$

where TP and TN denote the number of true positives and true negatives, respectively.

Precision is the proportion of predicted true-positive values to the total number of predicted true-positive and false-positive values. A model with a low precision is prone to a high false-positive rate. Precision can be calculated using the following equation:

(8) $$\begin{array}{c} \text{precision}=\frac{\text{TP}}{\text{FP}+\text{TP}}, \end{array}$$

where FP denotes the number of false positives.

The number of true positives divided by the sum of true positives and false negatives is known as recall or sensitivity. When there is a large cost associated with false negatives, the model statistic used to pick the optimal model is recall. Recall can be computed using the following equation:

(9) $$\begin{array}{c} \text{recall}=\frac{\text{TP}}{\text{TP}+\text{FN}}, \end{array}$$

where FN denotes the number of false negatives.

Specificity is the proportion of predicted true negatives to the summation of predicted true negatives and false positives. Specificity can be determined using the following equation:

(10) $$\begin{array}{c} \text{specificity}=\frac{\text{TN}}{\text{TN}+\text{FP}}. \end{array}$$

*F*_1_-score combines precision and recall. As a result, both false positives and false negatives are included while calculating this score. It is not as simple as accuracy for comparison. However, *F*_1_-score is generally more valuable than accuracy, particularly if the problem is an imbalanced classification problem. The following equation can be used to calculate the *F*_1_-score:

(11) $$\begin{array}{c} F_{1}-\text{score}=\frac{2\times \text{recall}\times \text{precision}}{\text{recall}+\text{precision}}. \end{array}$$

In this study, the dataset that Ozturk et al. [6] collected has been employed, gathered from two distinct sources, and includes COVID-19, No-findings, and Pneumonia, as shown in Figure 2. The first class of dataset contained 43 women, and 82 men confirmed they were infected with COVID-19. The average age of 26 COVID-19 confirmed individuals is about 55 years old, according to the age information supplied. The remaining two classes were chosen randomly from the Wang et al. [58] ChestX-ray8 dataset, including 500 No-findings and 500 Pneumonia images.

Two distinct perspectives were conducted to identify and classify COVID-19. First, the proposed technique was validated in order to classify two classes labeled COVID-19 and No-findings. Second, the proposed approach was used to classify three different groups: COVID-19, No-findings, and Pneumonia. In the first aspect, the two-class problem, the proposed method effectiveness is measured using the 5-fold cross-validation. A total of 80% of the dataset was used for training and 20% for testing. Following the extraction of features by DenseNet169, ANOVA selected 67 features from 1664 as an optimal number for classification, resulting in about 96% of features being reduced, and the XGBoost classification process was significantly sped up.

The 5-fold cross-validation had an average accuracy of 98.72%, and the confusion matrix was computed for each fold and overlapped, as shown in Figure 3. The confusion matrix entries acquired in all folds are used to generate the overlapping confusion matrix. It shows that the proposed architecture correctly identified COVID-19 and No-findings with 100% and 98.43% accuracy, respectively. In other words, the proposed method performs better at detecting true-positive samples.

The achieved precision, recall, specificity, and *F*_1_-score values were 99.21%, 93.33%, 100%, and 97.87%, respectively.  Table 1 represents the comparison of the proposed method with Ozturk et al. [6] and Nasiri and Hasani [21] in terms of accuracy, precision, recall, specificity, and *F*_1_-score values for each fold and the average of all folds, which Nasiri and Hasani [21] had better results than Ozturk et al. [6] and the proposed method outperforms them all except recall. The good performance of the proposed method can be attributed to the superiority of the XGBoost, which has a good generalization and less overfitting. As a result, the proposed method outperforms other methods in terms of test accuracy. Furthermore, using ANOVA helps the proposed method select the most distinctive features from the feature space and better separate COVID-19, No-findings, and Pneumonia classes, leading to higher classification accuracy.

In the multiclass problem, 80% of the X-ray images dataset was used for training, and the remaining 20% was employed as the test set. ANOVA was used to select 275 features out of 1664 as the ideal number for classification. Consequently, almost 84% of features were decreased, and XGBoost classification process was substantially ramped up, and performance improved. The accuracy on the test set was 92%. The confusion matrix is illustrated in Figure 4. Like two-class problem, this confusion matrix indicates that the proposed method had a better result in finding COVID-19 than No-findings and Pneumonia. Precision, recall, specificity, and *F*_1_-score values of 94.07%, 88.46%, 100%, and 92.42% were reached, respectively. Regarding accuracy, precision, recall, specificity, and *F*_1_-score values of the test set, Table 2 compares the proposed approach to Ozturk et al. [6] and Nasiri and Hasani [21].

The proposed method was applied to nine pretrained networks for both binary and multiclass problems. As shown in Table 3, the average of 5-fold cross-validation accuracy was employed to compare approaches in binary class problem, whereas the best fold accuracy was used to compare approaches on the multiclass problem. DenseNet169 outperforms other pretrained networks in both binary and multiclass problems. Additionally, the gradient-based class activation mapping (Grad-CAM) [59] was used to represent the decision area on a heatmap.  Figure 5 illustrates the heatmaps for three COVID-19 cases, confirming that the proposed method extracted correct features for detection of COVID-19, and the model is mostly concentrated on the lung area. Radiologists might use these heatmaps to evaluate the chest area more accurately.

The proposed method was compared to relevant works in Table 4. Gunraj et al. [8] applied 16,756 X-ray chest images from diverse sources to develop COVID-Net and achieved a 92.40% accuracy rate on the multiclass classification problem. Sethy et al. [27] reached 95.38% accuracy using ResNet50 and SVM, which was evaluated by 50 X-ray images. Wang et al. [30] proposed M-Inception for 195 COVID-19 infected patients and 258 healthy cases, and as a result, they achieved an 82.90% accuracy rate. Hemdan et al. [36] trained and evaluated COVIDX-Net using 25 confirmed COVID-19 and 25 noninfected cases X-ray images, achieving a 90.00% accuracy rate.

Narin et al. [33] used 50 public source COVID-19 chest X-ray images and 50 normal images from another source to test three alternative CNN models, obtaining a 98.00% accuracy rate. Song et al. [60] employed 777 confirmed COVID-19 patients and 708 normal cases CT images to develop their deep model based on the pretrained network model, ResNet50, which reached an 86.0% accuracy rate.

Zheng et al. [61] gained 90.80% accuracy employing CT images of 313 positive COVID-19 and 229 normal cases to develop their model. Xu et al. [35] applied ResNet on the dataset of 219 confirmed COVID-19 and 224 Pneumonia and 175 normal CT images, scoring 86.70% performance. Ozturk et al. [6] used 125 positive COVID-19, 500 No-findings, and 500 Pneumonia X-ray images to develop their model, resulting in 98.08% for two-class and 87.02% multiclass accuracy rate. The dataset that Ozturk et al. [6] gathered from various sources was used in this paper. For the two-class and multiclass classification problems, 98.72% and 92.00% accuracy rates were obtained, respectively, in this paper. Table 4 shows that the proposed approach outperforms most of the existing deep learning-based models in terms of accuracy. However, it should be emphasized that the findings in Table 4 were derived from different datasets and different experimental setups. This study's limitations and drawbacks include using a limited number of COVID-19 X-ray images (i.e., 125 samples) and sensitivity of the proposed method's performance to the number of features selected by ANOVA so that the number of features should be selected by trial and error.

## 5. Conclusion

Early diagnosis of COVID-19 is a crucial step to prevent mortality and transmission of the virus. RT-PCR is the most accessible tool to identify COVID-19, but finding other alternatives for this problem is essential due to false-negative outcomes and time limitations. Chest CT and X-ray images are suitable substitutes for RT-PCR, but because of the lack of CT hardware, X-ray images are a superior tool for diagnosing COVID-19. AI and machine learning-based methods play a crucial role in the quicker detection of COVID-19. In this study, a pretrained model, DenseNet169, was utilized to extract features from X-ray images, and ANOVA was employed to select features to decrease classification time and improve performance. Finally, selected features were classified using XGBoost. The ChestX-ray8 dataset was used to evaluate the proposed method. The proposed method reached 98.72% accuracy for the two-class problem and 92% accuracy for the multiclass problem. The proposed method's precision, recall, and specificity rates on the two-class problem were 99.21%, 93.33%, and 100%, respectively. Also, for the multiclass problem, the proposed method achieved 94.07% precision, 88.46% recall, and 100% specificity. The experimental results show that the proposed method outperforms other state-of-the-art methods, and radiologists might use it to detect COVID-19 cases more accurately.

## Figures and Tables

**Figure 1:** The architecture of the proposed model.

**Figure 2:** Representation of chests X-ray in COVID-19 patients (a), No-findings (b), and patients with Pneumonia (c).

**Figure 3:** Confusion matrix for the two-class problem.

**Figure 4:** Confusion matrix for the multiclass problem.

**Figure 5:** The heatmap of three confirmed COVID-19 X-ray images.

**Table 1:** Comparison of the proposed method with other methods in two-class problem.

Performance metrics (%)	Methods	1-fold	2-fold	3-fold	4-fold	5-fold	Average
Recall	Proposed method	94.73	90.47	92.00	**96.96**	92.59	93.33
	Ozturk et al.	**100**	**96.42**	90.47	93.75	**93.18**	**95.13**
	Nasiri and Hasani	95.20	95.40	**96.70**	81.40	91.40	92.08

Specificity	Proposed method	**100**	**100**	**100**	**100**	**100**	**100**
	Ozturk et al.	**100**	96.42	90.47	93.75	93.18	95.30
	Nasiri and Hasani	**100**	**100**	**100**	89.90	**100**	99.78

Precision	Proposed method	99.53	99.05	99.01	**99.46**	99.00	**99.21**
	Ozturk et al.	**100**	94.52	98.14	98.57	98.58	98.03
	Nasiri and Hasani	99.50	**99.50**	**99.40**	95.30	**99.02**	98.54

*F*_1_-score	Proposed method	98.41	97.02	97.42	**98.96**	**97.57**	**97.87**
	Ozturk et al.	**100**	95.52	93.79	95.93	95.62	96.51
	Nasiri and Hasani	98.50	**98.50**	**98.20**	92.50	97.30	97.00

Accuracy	Proposed method	99.20	98.40	98.40	**99.20**	**98.40**	**98.72**
	Ozturk et al.	**100**	97.60	96.80	97.60	97.60	98.08
	Nasiri and Hasani	99.20	**99.20**	**99.20**	95.20	**98.40**	98.24

**Table 2:** Comparison of the proposed method with other methods in multiclass problem.

Methods	Performance metrics (%)				
	Recall	Specificity	Precision	*F*_*1*_-score	Accuracy
Proposed method	88.46	**100**	**94.07**	**92.42**	**92.00**
Ozturk et al.	88.17	93.66	90.97	89.44	89.33
Nasiri and Hasani	**95.20**	**100**	92.50	91.20	89.70

**Table 3:** Comparison of different deep neural networks.

DNN	Binary class accuracy (%)	Multiclass accuracy (%)
DenseNet169	**98.72**	**92.00**
InceptionV3	92.96	82.22
NASNetLarge	94.88	84.00
ResNet152	94.71	77.33
VGG16	97.43	88.88
VGG19	97.28	88.88
Xception	95.68	80.88
EfficientNetB0	97.92	88.88
InceptionResNetV2	94.88	83.11

**Table 4:** Comparison of the proposed method with other DNN based methods.

Study	Type of images	Number of cases	Method used	Accuracy (%)	Drawbacks
Wang et al. [8]	Chest X-ray	358 COVID-19 (+)	COVID-Net	92.40	Use of an unbalanced dataset
		8066 COVID-19 (−)			High computational complexity due to training of deep neural network
		5538 Pneumonia			

Sethy et al. [27]	Chest X-ray	25 COVID-19 (+)	ResNet50 + SVM	95.38	Use of a dataset with a limited number of samples
		25 COVID-19 (−)			

Hemdan et al. [36]	Chest X-ray	25 COVID-19 (+)	COVIDX-Net	90.00	Use of a dataset with a limited number of samples
		25 COVID-19 (−)			

Narin et al. [33]	Chest X-ray	50 COVID-19 (+)	Deep CNN	98.00	Use of a dataset with a limited number of samples
		50 COVID-19 (−)	ResNet50		

Ying et al. [60]	Chest CT	777 COVID-19 (+)	DRE-Net	86.00	Low accuracy
		708 healthy			

Wang et al. [30]	Chest CT	195 COVID-19 (+)	M-Inception	82.90	Low accuracy
		258 COVID-19 (−)			

Zheng et al. [61]	Chest CT	313 COVID-19 (+)	UNet + 3D deep network	90.80	High computational complexity due to training of deep neural network
		229 COVID-19 (−)			

Xu et al. [35]	Chest CT	219 COVID-19 (+)	ResNet + location attention	86.70	Low accuracy
		224 viral pneumonia			High computational complexity due to training of deep neural network
		175 healthy			

Ozturk et al. [6]	Chest X-ray	125 COVID-19 (+)	DarkCovidNet	98.08	Use of a limited number of COVID-19 samples
		500 No-Findings			
		125 COVID-19 (+)		87.02	High computational complexity due to training of deep neural network
		500 No-Findings			
		500 Pneumonia			

Proposed method	Chest X-ray	125 COVID-19 (+)	DenseNet169+ ANOVA + XGBoost	**98.72**	Sensitivity to the number of features selected by the ANOVA
		500 No-Findings			
		125 COVID-19 (+)		**92.00**	Use of a limited number of COVID-19 samples
		500 No-Findings			
		500 Pneumonia			

## Data Availability

Publicly available ChestX-ray8 dataset was used in this study. The source code of the proposed method required to reproduce the predictions and results is available at https://github.com/seyyedalialavi2000/COVID-19-detection.

## References

[1] Khan A. I., Shah J. L., Bhat M. M. (2020). CoroNet: a deep neural network for detection and diagnosis of COVID-19 from chest x-ray images. *Computer Methods and Programs in Biomedicine*.

[2] Wu Z., McGoogan J. M. (2020). Characteristics of and important lessons from the coronavirus disease 2019 (COVID-19) outbreak in China. *JAMA*.

[3] Manoj M., Srivastava G., Somayaji S. R. K., Gadekallu T. R., Maddikunta P. K. R., Bhattacharya S. An incentive based approach for COVID-19 planning using blockchain technology.

[4] Bhattacharya S., Reddy Maddikunta P. K., Pham Q.-V. (2021). Deep learning and medical image processing for coronavirus (COVID-19) pandemic: a survey. *Sustainable Cities and Society*.

[5] Fronstin P., Woodbury S. A. (2020). *How Many Americans Have Lost Jobs with Employer Health Coverage During the Pandemic*.

[6] Ozturk T., Talo M., Yildirim E. A., Baloglu U. B., Yildirim O., Rajendra Acharya U. (2020). Automated detection of COVID-19 cases using deep neural networks with X-ray images. *Computers in Biology and Medicine*.

[7] Bhatt T., Kumar V., Pande S., Malik R., Khamparia A., Gupta D. (2021). A review on COVID-19. *Artificial Intelligence and Machine Learning for COVID-19*.

[8] Gunraj H., Wang L., Wong A. (2020). COVIDNet-CT: a tailored deep convolutional neural network design for detection of COVID-19 cases from chest CT images. *Frontiers of Medicine*.

[9] Tabik S., Gomez-Rios A., Martin-Rodriguez J. L. (2020). COVIDGR dataset and COVID-SDNet methodology for predicting COVID-19 based on chest X-ray images. *IEEE Journal of Biomedical and Health Informatics*.

[10] Huang P., Liu T., Huang L. (2020). Use of chest CT in combination with negative RT-PCR assay for the 2019 novel coronavirus but high clinical suspicion. *Radiology*.

[11] Ai T., Yang Z., Hou H. (2020). Correlation of chest CT and RT-PCR testing for coronavirus disease 2019 (COVID-19) in China: a report of 1014 cases. *Radiology*.

[12] Ahishali M., Degerli A., Yamac M. (2021). Advance warning methodologies for COVID-19 using chest x-ray images. *IEEE Access*.

[13] Ilyas M., Rehman H., Nait-Ali A. (2020). Detection of Covid-19 from chest X-ray images using artificial intelligence: an early review. https://arxiv.org/abs/2004.05436.

[14] Fang Y., Pang P. (2020). Senivity of chest CT for COVID-19: comparasion to RT-PCR. *Radiology*.

[15] Xie X., Zhong Z., Zhao W., Zheng C., Wang F., Liu J. (2020). Chest CT for typical coronavirus disease 2019 (COVID-19) pneumonia: relationship to negative RT-PCR testing. *Radiology*.

[16] Shi F., Wang J., Shi J. (2020). Review of artificial intelligence techniques in imaging data acquisition, segmentation, and diagnosis for COVID-19. *IEEE Reviews in Biomedical Engineering*.

[17] Zhu N., Zhang D., Wang W. (2020). A novel coronavirus from patients with pneumonia in China, 2019. *New England Journal of Medicine*.

[18] Lecun Y., Bengio Y., Hinton G. (2015). Deep learning. *Nature*.

[19] Nasiri H., Alavi S. A. (2021). A novel framework based on deep learning and anova feature selection method for diagnosis of COVID-19 cases from chest X-ray images. https://arxiv.org/abs/2110.06340.

[20] Apostolopoulos I. D., Mpesiana T. A. (2020). COVID-19: automatic detection from x-ray images utilizing transfer learning with convolutional neural networks. *Physical and Engineering Sciences in Medicine*.

[21] Nasiri H., Hasani S. (2021). Automated detection of COVID-19 cases from chest X-ray images using deep neural network and XGBoost. https://arxiv.org/abs/2109.02428.

[22] Qaid T. S., Mazaar H., Al-Shamri M. Y. H., Alqahtani M. S., Raweh A. A., Alakwaa W. (2021). Hybrid deep-learning and machine-learning models for predicting COVID-19. *Computational Intelligence and Neuroscience*.

[23] Abdulkareem K. H., Mohammed M. A., Salim A. (2021). Realizing an effective COVID-19 diagnosis system based on machine learning and IoT in smart hospital environment. *IEEE Internet of Things Journal*.

[24] Chen L., Rezaei T. (2021). A new optimal diagnosis system for coronavirus (COVID-19) diagnosis based on Archimedes optimization algorithm on chest X-ray images. *Computational Intelligence and Neuroscience*.

[25] Khorami E., Mahdi Babaei F., Azadeh A. (2021). Optimal diagnosis of COVID-19 based on convolutional neural network and red Fox optimization algorithm. *Computational Intelligence and Neuroscience*.

[26] Waheed A., Goyal M., Gupta D., Khanna A., Al-Turjman F., Pinheiro P. R. (2020). CovidGAN: data augmentation using auxiliary classifier GAN for improved covid-19 detection. *IEEE Access*.

[27] Sethy P. K., Behera S. K., Ratha P. K., Biswas P. (2020). Detection of coronavirus disease (COVID-19) based on deep features and support vector machine. *International Journal of Mathematical, Engineering and Management Sciences*.

[28] Ahmad F., Farooq A., Ghani M. U. (2021). Deep ensemble model for classification of novel coronavirus in chest X-ray images. *Computational Intelligence and Neuroscience*.

[29] Abbas A., Abdelsamea M. M., Gaber M. M. (2021). Classification of COVID-19 in chest X-ray images using DeTraC deep convolutional neural network. *Applied Intelligence*.

[30] Wang W., Li Y., Wang X., Li J., Zhang P. COVID-19 patients detection in chest X-ray images via MCFF-net.

[31] Ucar F., Korkmaz D. (2020). COVID diagnosis-Net: deep Bayes-SqueezeNet based diagnosis of the coronavirus disease 2019 (COVID-19) from X-ray images. *Medical Hypotheses*.

[32] Wang S., Kang B., Ma J. (2021). A deep learning algorithm using CT images to screen for Corona Virus Disease (COVID-19). *European Radiology*.

[33] Narin A., Kaya C., Pamuk Z. (2020). Department of biomedical engineering, zonguldak bulent ecevit university, 67100. https://arxiv.org/abs/2003.10849.

[34] He X., Yang X., Zhang S. (2020). Sample-efficient deep learning for COVID-19 diagnosis based on CT scans. *IEEE Transactions on Medical Imaging*.

[35] Xu X., Jiang X., Ma C. (2020). A deep learning system to screen novel coronavirus disease 2019 pneumonia. *Engineering*.

[36] Hemdan E. E.-D., Shouman M. A., Karar M. E. (2020). Covidx-net: a framework of deep learning classifiers to diagnose COVID-19 in x-ray images. https://arxiv.org/abs/2003.11055.

[37] Minaee S., Kafieh R., Sonka M., Yazdani S., Jamalipour Soufi G. (2020). Deep-COVID: predicting COVID-19 from chest X-ray images using deep transfer learning. *Medical Image Analysis*.

[38] Adnan M., Rahman F., Imrul M., AL N., Shabnam S. (2018). Handwritten bangla character recognition using inception convolutional neural network. *International Journal of Computer Application*.

[39] Lecun Y., Bottou L., Bengio Y., Haffner P. (1998). Gradient-based learning applied to document recognition. *Proceedings of the IEEE*.

[40] Zhou P., Ni B., Geng C., Hu J., Xu Y. Scale-transferrable object detection. *CVF Open Access*.

[41] Huang G., Liu Z., Van Der Maaten L., Weinberger K. Q. Densely connected convolutional networks.

[42] Chandrashekar G., Sahin F. (2014). A survey on feature selection methods. *Computers & Electrical Engineering*.

[43] Guyon I., Elisseeff A. (2003). An introduction to variable and feature selection. *Journal of Machine Learning Research*.

[44] Johnson K. J., Synovec R. E. (2002). Pattern recognition of jet fuels: comprehensive GC × GC with ANOVA-based feature selection and principal component analysis. *Chemometrics and Intelligent Laboratory Systems*.

[45] Lin H., Ding H. (2011). Predicting ion channels and their types by the dipeptide mode of pseudo amino acid composition. *Journal of Theoretical Biology*.

[46] Ding H., Guo S.-H., Deng E.-Z. (2013). Prediction of Golgi-resident protein types by using feature selection technique. *Chemometrics and Intelligent Laboratory Systems*.

[47] Chen T., Guestrin C. Xgboost: a scalable tree boosting system.

[48] Chelgani S. C. (2021). Estimation of gross calorific value based on coal analysis using an explainable artificial intelligence. *Machine Learning with Applications*.

[49] Song K., Yan F., Ding T., Gao L., Lu S. (2020). A steel property optimization model based on the XGBoost algorithm and improved PSO. *Computational Materials Science*.

[50] Chehreh Chelgani S., Nasiri H., Tohry A. (2021). Modeling of particle sizes for industrial HPGR products by a unique explainable AI tool- A “Conscious Lab” development. *Advanced Powder Technology*.

[51] Chelgani S. C., Nasiri H., Alidokht M. (2021). Interpretable modeling of metallurgical responses for an industrial coal column flotation circuit by XGBoost and SHAP-A ‘conscious-lab’ development. *International Journal of Mining Science and Technology*.

[52] Zhang D., Chen H.-D., Zulfiqar H. (2021). IBLP: an XGBoost-based predictor for identifying bioluminescent proteins. *Computational and Mathematical Methods in Medicine*.

[53] Nasiri H., Homafar A., Chelgani S. C. (2021). Prediction of uniaxial compressive strength and modulus of elasticity for Travertine samples using an explainable artificial intelligence. *Results in Geophysical Sciences*.

[54] Yu B., Qiu W., Chen C. (2020). SubMito-XGBoost: predicting protein submitochondrial localization by fusing multiple feature information and eXtreme gradient boosting. *Bioinformatics*.

[55] Lin M., Chen Q., Yan S. Network in network.

[56] Tang J., Alelyani S., Liu H. (2014). Feature selection for classification: a review. *Data Classification Algorithms and Applications*.

[57] Maxwell A., Li R, Yang B (2017). Deep learning architectures for multi-label classification of intelligent health risk prediction. *BMC Bioinformatics*.

[58] Wang X., Peng Y., Lu L., Lu Z., Bagheri M., Summers R. M. Chest x-ray 8: hospital-scale chest x-ray database and benchmarks on weakly-supervised classification and localization of common thorax diseases.

[59] Selvaraju R. R., Cogswell M., Das A., Vedantam R., Parikh D., Batra D. Grad-cam: visual explanations from deep networks via gradient-based localization.

[60] Song Y., Zheng H., Li L. (2021). Deep learning enables accurate diagnosis of novel coronavirus (COVID-19) with CT images. *IEEE/ACM Transactions on Computational Biology and Bioinformatics*.

[61] Zheng C., Deng X., Fu Q., Zhou Q (2020). Deep learning-based detection for COVID-19 from chest CT using weak label. *MedRxiv*.

